# Fractal Characteristics of May-Grünwald-Giemsa Stained Chromatin Are Independent Prognostic Factors for Survival in Multiple Myeloma

**DOI:** 10.1371/journal.pone.0020706

**Published:** 2011-06-16

**Authors:** Daniela P. Ferro, Monica A. Falconi, Randall L. Adam, Manoela M. Ortega, Carmen P. Lima, Carmino A. de Souza, Irene Lorand-Metze, Konradin Metze

**Affiliations:** 1 Department of Pathology, University of Campinas, Campinas, Brazil; 2 Hematology/Hemotherapy Center, University of Campinas, Campinas, Brazil; 3 Department of Internal Medicine, University of Campinas, Campinas, Brazil; 4 Institute of Computing, University of Campinas, Campinas, Brazil; Roswell Park Cancer Institute, United States of America

## Abstract

**Background:**

The use of computerized image analysis for the study of nuclear texture features has provided important prognostic information for several neoplasias. Recently fractal characteristics of the chromatin structure in routinely stained smears have shown to be independent prognostic factors in acute leukemia. In the present study we investigated the influence of the fractal dimension (FD) of chromatin on survival of patients with multiple myeloma.

**Methodology:**

We analyzed 67 newly diagnosed patients from our Institution treated in the Brazilian Multiple Myeloma Study Group. Diagnostic work-up consisted of peripheral blood counts, bone marrow cytology, bone radiograms, serum biochemistry and cytogenetics. The International Staging System (ISS) was used. In every patient, at least 40 digital nuclear images from diagnostic May-Grünwald-Giemsa stained bone marrow smears were acquired and transformed into pseudo-3D images. FD was determined by the Minkowski-Bouligand method extended to three dimensions. Goodness-of-fit of FD was estimated by the R^2^ values in the log-log plots. The influence of diagnostic features on overall survival was analyzed in Cox regressions. Patients that underwent autologous bone marrow transplantation were censored at the day of transplantation.

**Principal Findings:**

Median age was 56 years. According to ISS, 14% of the patients were stage I, 39% were stage II and 47% were stage III. Additional features of a bad prognosis were observed in 46% of the cases. When stratifying for ISS, both FD and its goodness-of-fit were significant prognostic factors in univariate analyses. Patients with higher FD values or lower goodness-of-fit showed a worse outcome. In the multivariate Cox-regression, FD, R^2^, and ISS stage entered the final model, which showed to be stable in a bootstrap resampling study.

**Conclusions:**

Fractal characteristics of the chromatin texture in routine cytological preparations revealed relevant prognostic information in patients with multiple myeloma.

## Introduction

Multiple myeloma (MM) is a clonal proliferation of malignant plasma cells characterized by a very heterogeneous disease outcome, varying from relatively asymptomatic slowly progressing forms to a frankly aggressive course. Moreover, important variations in tumor cell biology have been described, thus revealing a heterogeneous disorder [1]. In 2005 the International Staging System (ISS) was introduced, based on the serum concentrations of ß2-microglobulin and albumin, which provide prognostic stratification of the patients [1]–[5]. However, patient's age, degree of anemia, serum creatinine and calcium levels, dehydrogenase activity (LDH) as well as cytogenetic abnormalities have been described as additional prognostic factors [1], [3], [5]. Plasma cell morphology has also been recognized as an independent prognostic factor for more than two decades [1], [6]. However, the recognition of prognostically relevant cell atypias and maturation of the neoplastic plasma cells is dependent on the morphologist's expertise, thus leading to a considerable inter-observer variability. On the other hand, experimental studies using computerized image analysis have shown that subvisible modifications of the chromatin architecture in myeloma cells are associated with important changes of cell physiology, such as acquired drug resistance [7]. The quantitative analysis of the distribution pattern of chromatin and other nuclear components has been shown to be of prognostic importance in several neoplasias [8]–[15]. Therefore, we would expect that chromatin texture features in myeloma cells might reveal characteristics related to the aggressiveness of the tumor.

Scale-invariant self-similarity is an important feature of many biological structures. It cannot be described adequately by classic Euclidean geometry, but may be estimated by the determination of the fractal dimension. There is increasing use of fractal geometry for medical signal analysis with applications to pattern recognition, texture analysis and segmentation [16]–[25]. This analysis has also been applied for the study of cell nuclei, as the fractal nature of chromatin and its surrounding nucleoplasmic space has been demonstrated by different methods [26]–[28]. Moreover, the fractal characteristics of nuclear chromatin measured in cytological or histological preparations have shown to be of prognostic importance in several neoplasias [10], [13], [14], [28]–[33].

Therefore we investigated whether the fractal dimension of nuclear chromatin measured in routinely stained cytological smears of myeloma patients has a relation to the survival of the patients.

## Methods

### Study subjects

We analyzed retrospectively consecutive newly diagnosed patients with multiple myeloma treated at our Institution, where clinical data, diagnostic bone marrow (BM) smears, and cytogenetic analyses were available. The study was approved by the Ethics Committee of the Faculty of Medical Sciences, University of Campinas (process 365/2002). Patients gave written informed consent for participation in the study.

MM was diagnosed using the criteria of the International Myeloma Working Group, based on serum protein electrophoresis, presence of proteinuria, bone marrow cytology and bone radiograms [34]. The data about peripheral blood (PB) counts, bone marrow cytology, bone radiograms, serum biochemistry (calcium, albumin, creatinine and beta-2-microglobulin) and cytogenetics were recorded. Only patients that fulfilled the criteria for chemotherapy were included. Those with asymptomatic (smoldering) myeloma, immunoglobulin IgM–related disorders or with primary amyloidosis were excluded.

Staging was performed according to the ISS [2]. Moreover, using the criteria of Greipp et al [2], patients were classified as belonging to the very poor prognosis group, if one or more of the following criteria were fulfilled: serum ß2-microglobulin >10 mg/L, serum creatinine >4 mg/dL, serum albumin <2.5 g/dL, and platelet count <130×10^9^/l.

Cytogenetics had been performed in the diagnostic BM according to the method of Brigadeau et al [35]. In brief, BM nucleated cells were obtained by Ficoll-Hypaque centrifugation of the aspirated material. They were cultured for 72 hours in RPMI1640 supplemented with fetal calf serum. Cultures were performed both without stimulation, and with stimulation by IL-6 and GM-CSF. G-banding was analyzed, chromosome number and specific abnormalities were recorded.

Furthermore we looked for the presence of unfavorable cytogenetic alterations, such as hypodiploidy, deletion of chromosome 13, t(4;14), t(14:16), or 17p–, and counted for each patient the number of cytogenetic abnormalities.

The patients had been treated according to the Brazilian Multiple Myeloma Study Group [36] which consisted of an induction chemotherapy with VAD (vincristine 0.4 mg IV day 1, doxorubicin 9 mg/m^2^ IV day 1 and oral dexamethasone 40 mg daily), stem cell mobilization with cyclophosphamide (4 g/m^2^ IV), autologous bone marrow transplantation, and then randomized to test the utility for post-transplantation maintenance treatment using thalidomide.

Survival was measured from the diagnosis to time of death or last follow-up. Patients that underwent autologous bone marrow transplantation were censored at the day of transplantation.

### Morphometry

May-Grünwald-Giemsa stained bone marrow slides made at diagnosis were retrieved from the files. Neoplastic plasma cells were acquired in 24-bit color bitmap format with a Leica DC 500 (tm) digital camera (resolution of 12 megapixels, oil immersion objective ×100).

Randomly chosen, non-overlapping tumor nuclei were captured, interactively segmented and then converted to 8 bit gray scale with levels of luminance ranging between 0 and 255 (Fig. 1). For each nucleus, classical morphometric parameters such as nuclear area and the circular form factor (the ratio between perimeter of a circle with the same area as the nucleus and the actual nuclear perimeter) were calculated. In addition, the fractal dimension of each nucleus was determined.

**Figure 1:** Segmented nucleus (left) of a myeloma cell and its pseudo 3D transformation (middle). On the right side, the log-log-plot for the determination of the fractal dimension (FD), which is calculated from the slope of the ideal regression line (black) obtained by curve fitting. X-axis shows the logarithms of the inverse values of the size of the structuring element and y axis the logarithmic values of the fractal areas. (compare with the main text). R^2^ represents the goodness-of-fit of the real values (red), when compared with ideal regression line (black) and can be interpreted as a measure of “fractal quality”.

The fractal dimension of an object is, in many studies, measured after binarization of the image. Since we were dealing with 256 gray levels, binarization would be arbitrary and reduce the information content [10], [37], [38]. Therefore we decided not to binarize, but to apply the Minkowski-Bouligand method extended to pseudo-3D images [10], [39], [40], [41]. We created landscape-like pseudo-3D images, where the x and y coordinates represented the position of the pixel, and the z coordinate, its grey level (Fig. 1). The fractal dimension (FD) of the surface of the pseudo- 3-D images was calculated using a software developed in house by our group. In brief, we calculated the fractal area which is estimated by the volume/2e with e being the radius, varying between 1 and 30 pixels, of the non-planar structuring element in form of a ball. Then, we calculated the linear regression in a log-log plot of the fractal area versus e, with each plot containing 30 points (Fig. 1).We rotated the point distribution so that the slope was at 45 degrees. Then, the coefficient of the regression between the real and the estimated values was calculated [40], [41]. This R^2^ value characterizes the goodness-of-fit of the regression line and is therefore an estimate of the “quality of fractality”. An ideal fractal has a R^2^ = 1.0. The real fractals have R^2^ values <1.0 [41].

In a preliminary study we have found that the cumulative histograms for FD distribution in individual cases stabilized after examination of 25–35 cells (Fig. 2). Therefore, we decided to acquire at least 40 cells per smear.

**Figure 2:** Mean fractal dimension as a function of the number of nuclei examined in an individual case. The mean value stabilized after examination of 30–40 cells.

Finally, the prognostic relevance of all these parameters was analyzed in univariate and multivariate Cox regressions (p = 0.05 for input and p = 0.1 for output, backward conditional step-wise selection). The stability of the Cox model was tested by bootstrap resampling. This is a useful procedure to test the internal stability of a model proposed. It consists of creating new data sets of equal size by random sampling of the original data with replacement. In an individual new bootstrap sample, a patient may be represented once, multiple times or not at all. A new Cox regression (with the same conditions as in the original data set) was then calculated for each of these new data sets in order to obtain the bootstrap parameter estimates. This procedure is very useful in order to point out the most important variables [42], [43]. SPSS 8.0 and WinStat software were used for calculations.

In order to facilitate the comparison with previous studies that used plasma cell morphology, we randomly selected 107 nuclear images from our whole data pool and classified them in four categories (Fig. 3) A: Nuclei with a mature chromatin structure; B: immature nuclei with a less organized chromatin; C: Nuclei with a loose chromatin and a large nucleolus; and D: Nuclei with irregular and disorganized chromatin with many dark and light spots. Then we compared the FDs and R^2^ values between the four groups by analysis of variance followed by the least square difference post-hoc test. Differences were considered significant when p<0.05.

**Figure 3:** Segmented images of myeloma cell nuclei, classified by their grade of maturity and chromatin structure. A: Nucleus with a more mature chromatin structure; its FD was 2.074935 and R^2^ = 0.999330. B: a more immature nucleus with a less organized chromatin structure presenting FD = 2.223 and R^2^ = 0.99896. C: Nucleus with a blastic feature: FD = 2.1759 and R^2^ = 0.9961. D: Nucleus with irregular and disorganized chromatin: FD = 2.2629 and R^2^ = 0.99931

## Results

Sixty seven patients entered the study: 39 men and 28 women. The clinical data are shown on table 1. Median age was 56 years. According to ISS there was a predominance of advanced cases. Additional features of a very bad prognosis were found in 46% of the patients. Among them, a β2-microglobulin value >10 mg/L was found in 37%, platelets were <130×10^9^/L in 21%, creatinine was >4 mg/dL in 15% and albumin was <2.5 g/dL in 19% of the patients. The mean follow-up was 25.4 months (1–227). At the end of the observation period 36 patients had died from multiple myeloma, 24 of them before having completed the VAD regimen.

**Table 1:** Clinical variables of the patients.

Variables	Median and range
Age (years)	56 (30–85)
ISS Stage I	10 (14%)
ISS stage II	26 (39%)
ISS stage III	31 (47%)
Hemoglobin g/dL	9.2 (3.5–14.5)
Leukocytes ×10^9^/l	6.1 (1.8–28.2)
Platelets ×10^9^/l	211 (16–580)
β2-microglobulin (mg/dL)	10.3 (1.7–290.0)
Creatinine (mg/dL)	1.3 (0.2–6.8)
Albumin g/dL	3.3 (1.1–5.8)
Calcium (mg/dL)	9.3 (6.7–16.3)

ISS (Fig. 4) was a significant adverse prognostic factor in the univariate Cox regression (stage I: B = −2.30; stage II B = −1.50; stage III: B = 0.0; p = 0.002). Patients belonging to the very poor prognostic group had a significant shorter survival (median 12.1 months) than all other patients (median 101.6 months) (B = 0.7562; p = 0.0302) (Fig. 5).

**Figure 4:** Overall survival of the myeloma patients categorized by ISS stage. Kaplan-Meier plot. Log rank-test: p = 0.0005.

**Figure 5:** Overall survival categorized by the presence or absence of additional risk factors [2]. Kaplan-Meier plot. Log rank-test: p = 0.02.

Age, serum calcium concentration, hemoglobin value, PB platelet count, BM percentage of myeloma cells, nuclear area and form factor had no prognostic relevance.

The morphometric features studied are shown in table 2. The fractal dimension (FD) was an adverse prognostic feature (B = 12.33; p = 0.0287). Only in order to illustrate the importance of FD as a prognostic variable, we dichotomized the continuous variable FD according to a cluster analysis (Ward algorithm), which suggested as cut-point at FD = 2.13 and then created a Kaplan-Meier-plot (Fig. 6). The goodness-of -fit (R^2^) was a favorable prognostic factor in the univariate Cox regression when stratified for ISS (B = −592.6; p = 0.10) (table 3).

**Figure 6:** Survival of the patients grouped by FD. Kaplan-Meier plot. Log rank-test: p = 0.05.

**Table 2:** Morphometric variables of the nuclei of the myeloma cells.

Variables	Median and range
Nuclear area (µm^2^)	64.0 (42.1–99.7)
Form factor	0.5195 (0.4362–0.5651)
FD Minkowski	2.113 (2.071–2.278)
R^2^	0.99875 (0.99642–0.99997)

**Table 3:** Factors influencing the survival of the patients, analyzed by the univariate Cox regression.

	B	p
ISS stage l	−2.30	0.001
ISS stage II	−1.50	0.025
ISS stage III	0.00	0.001
Very poor prognostic group	0.756	0.03
Cytogenetics	0.883	0.038
FD Minkowski	12.33	0.028
R ^2^ (stratified by ISS)	−592.6	0.10

Cytogenetic analysis revealed hyperdiploidy in 12 cases, alterations of chromosome 13 in 2 patients, 2 cases with translocations involving chromosome 14 (in one case together with −17) and 1 patient with hypodiploidy. The number of cytogenetic abnormalities was an adverse prognostic factor in the univariate Cox regression (B = 0.8833; p = 0.0387).

The nuclear area, form factor, FD and goodness-of-fit did not correlate with ISS stage or laboratory parameters, such as serum calcium concentration, β2-microglobulin, albumin, creatinine, hemoglobin value, PB platelet count and BM percentage of myeloma cells (Spearman rank order test). We could not detect any statistical relation between presence or number of chromosomal abnormalities and FD (Spearman rank order correlation).

Looking at the morphology of the neoplastic plasma cell nuclei (Fig. 3), mature plasma cells showed significantly the lowest fractal dimension (FD = 2.08) whereas the FDs of all other cell types were significantly higher (FD immature  = 2.15; FD blasts  = 2.18 and FD irregular nuclei  = 2.16). There was, however, no statistically significant difference between these three cell types. Goodness-of-fit was significantly lowest for cells with irregular nuclei (R^2^ = 0.9978), followed by blasts (R^2^ = 0.9987). Mature (0.9993) and immature (0.9993) plasma cells revelaed significantly the highest values, yet without any difference between them.

Finally, all variables with p≤0.10 in the univariate analyses (ISS, very poor risk group, FD, R^2^ FD and cytogenetic alterations) were simultaneously analyzed in a multivariate proportional hazard model. The final Cox regression included ISS (stage I: B = −2.13; stage II: B = −1.75; stage III: B = 0.0; p = 0.0004), FD (B = 14.39; p = 0.015), R^2^ FD (B = −935.12; p = 0.0317) and the number of genetic alterations (B = 0.8862; p = 0.069), whereas the variable “very poor prognosis group” did not enter the model.

The stability of this model was confirmed in a bootstrap resampling procedure. Among 100 new models, “ISS” entered in 100%, “fractal dimension” in 77%, “R^2^ FD” in 68%, “number of cytogenetic abnormalities” in 60%, but “very poor prognosis group” entered in none of the models.

## Discussion

The median age of our patients at diagnosis was 56 years, which is considerably lower than that reported in studies on MM from North America, Europe or Asia [2], [44]. A younger age of the patients at diagnosis, when compared with other countries, has also been reported for other hematological neoplasias in Brazil, such as myelodysplastic syndromes and myeloid leukemias [45]–[51]. Besides that, a recent epidemiological survey of patients with multiple myeloma in our country showed a similar mean age and also a high frequency of advanced ISS [45]. No final conclusive explanation has been found for this phenomenon. But one might speculate that this could be due to a high exposure to carcinogenic agents in Brazil. It has been shown that herbicides and pesticides are risk factors for the genesis of multiple myeloma [52]. But not only farm workers with direct contact to these toxins are at risk. The general population may be frequently exposed to residual toxins in food [53], [54].

Our patients showed a high frequency of advanced disease according to the ISS and additional poor risk factors. This resulted in a median survival of 24.9 months for all patients, much shorter than that reported by other studies [2], [45]. There are several possible explanations for this phenomenon. Delayed diagnosis in patients who depend on a public health system, as in our case, is not rare. In addition, unawareness of symptoms or indolence might be common in patients from lower socio-economic classes. And finally, a more aggressive character of MM in our country cannot be totally excluded. The patients with additional poor prognostic factors had a median survival of about 12.1 months, which is close to that reported by Greipp at al [2]. However, only 5% of the total population reported in that study had these criteria for additional high risk.

The International Staging System (ISS), based only on two laboratory variables, the β2-microglobulin and albumin serum concentrations, has replaced the Durie-Salmon staging system in 2005 and is currently considered standard for staging of myeloma [2], [5], [51]. It was further validated in patients in North America, Europe, and Asia; in patients below and above 65 years of age; in patients with standard therapy or autologous bone marrow transplantation; and in comparison with the Durie/Salmon staging system. The prognostic importance of this staging system was confirmed in our study.

Regarding the great variability of myeloma pathophysiology, there are additional prognostic factors, such as age, hemoglobin concentration, serum creatinine and calcium levels. But, this could not be confirmed in our investigation. Since the number of patients was relatively small, the test power was limited and we may have missed to demonstrate them as significant risk factors. Special attention was drawn to prognostic factors, which could improve a risk-stratification model able to define high-risk patients who can benefit from novel therapeutic strategies.

Plasma cell cytogenetic abnormalities and labeling index have also shown to be of prognostic value, but, these techniques require fresh unfixed material, are sophisticated and expensive, and can be performed only in few laboratories. Therefore it would be interesting to look for additional prognostic factors, which are not cost-expensive, can be examined retrospectively and be assessed independently of a specialized laboratory.

Cell morphology, evaluated subjectively by a trained observer, has also been considered a prognostic variable in multiple myelomas [6] but the drawback of this method is the considerable inter-observer variability. Goasguen et al. developed a protocol for morphologic analysis of myeloma cells based on more objective morphologic criteria in routinely stained slides [6]. These criteria included the presence of a nucleolus, blast-like chromatin and a nuclear-cytoplasmatic ratio >0.6, thus creating 8 possible subtypes. This procedure was able to identify an intermediate prognostic subgroup of patients, but the method was still dependent on a trained human observer [6]. Leleu et al [1] described in detail the nuclear shape changes in myeloma cells and created the variable “percentage of plasma cells with irregular nuclear shape”. This variable was a prognostic factor in the univariate analysis and significantly associated with other prognostic parameters such as Ki67 labeling index, hemoglobin values and hypodiploidy, but not with beta-2-microglobulin. In both studies, however, morphologic variables were not independent risk factors in multivariate regressions.

Computerized analysis of microscopic images overcomes the necessity of morphologic expertise and expert opinion and has shown to be an objective and reproducible method for diagnostic and prognostic purposes [33], [55]–[57]. Image analysis is able to detect subtle morphologic changes which cannot be recognized even by a trained observer [23], [56]–[58]. Among these techniques, the examination of the fractal characteristics of nuclear chromatin has shown to be of increasing importance [59]–[64].

The use of the fractal concept for image analysis has several advantages. The fractal dimension has shown to be robust against the segmentation process [63]. In routine cytological preparations fractal derived variables are much less dependent on staining variations than variables derived from the grey-level co-occurrence matrix [61]. Form factors, which are classically used for the quantitative description of irregular outlines, depend highly on the magnification scale, whereas fractals are scale independent [62].

The fractal dimension represents a statistical description but, moreover, is also intimately related to the theoretical concepts of complexity and morphogenesis. Therefore it provides a deeper insight into the understanding of the biology of normal tissues and neoplasias [16], [28]. The fractal concept, developed by Mandelbrot [64] in the sixties and seventies of the last century got popularity due to the famous images created by computer programs based on fractal geometry. It is however a ubiquitous theoretical framework for many processes or objects in our known universe. Fractality implies scale-independent self-similarity or self-affinity. The fractal concept may be applied to every kind of science. Fractal characteristics can be found when measurement values of a certain variable are scale independent so that in a log-log plot the measurement points can be well approximated by a regression line. Therefore the fractal property is always related to a measurement variable. An “object” or a “process” can reveal simultaneously fractal characteristics of many different variables or features.

Introducing the fractal concept in biology and medicine has improved our understanding of many physiological processes, such as allometric scaling growth, allosteric enzyme kinetics, intracellular bio-energetic dynamics, metabolic rate in mammals, population genetics, modeling of drug clearance, neo-angiogenesis, tumor growth, organization of nucleotides in DNA and RNA, and cardiovascular physiology [16], [18], [21], [65]–[68]. Fractals are very useful to characterize properly the complexity of macroscopic and microscopic anatomy, namely to describe the design principles underlying living organisms.

The chromatin structure can also be analyzed by fractal geometry [10], [14], [16], [17], [22], [23], [63]–[68].

Fractal structures can be created by iterations [69]. This happens for instance during condensation of a polymer such as DNA when it is repeatedly subjected to the self-similar process of crumpling. The result is a folded polymer with fractal properties. In this way, a long polymer can be packed in a small volume without entanglements. This facilitates unravelling when necessary, as for DNA transcription, and is therefore advantageous for cell physiology [68]. Recent studies using different methods of analysis showed that DNA, nuclear chromatin and the surrounding nucleoplasmic space have a fractal organization [26]–[28], [68],

Our study revealed that the staining pattern of nuclear chromatin of myeloma cells, (May-Grünwald –Giemsa method) has also fractal characteristics. An important challenge is to explain, why patients with a worse prognosis, revealed an increased FD of the chromatin staining pattern in May-Grünwald –Giemsa stained smears. Changes of the nuclear architecture, observed in histological or cytological preparations, reflect genomic and non-genomic alterations.

Multiple genetic aberrations have been described during the pathogenesis of multiple myelomas [70]. Secondary translocations and gene mutations have been implicated in disease progression, such as complex abnormalities of MYC, activation of N-RAS, K-RAS, and FGFR3 mutations, mutations or deletions of TP53, RB1, and PTEN and inactivation of cyclin-dependent kinase inhibitors [71], [72].

Furthermore, epigenetic changes causing altered gene and protein expression play a major role in the pathogenesis of multiple myelomas. Hypermethylation of the genes p15, p16, DAP-kinase, BAD, BAK, BAX, BIK, SOCS-1, and E-Cadherin, has been reported [71], [72].

Hypermethylation of CpG islands within gene promoter regions accompanied by deacetylation of histone proteins provokes transcriptional silencing. In parallel, global hypomethylation of repetitive elements occurs in association with tumor progression and increase of chromosomal instability [71], [72]. Therefore, in advanced cases, which are genetically unstable and therefore more aggressive, we expect a more complex chromatin rearrangement with global hypomethylaton and an increased number of hypermethylated CPG islands.

The routinely MGG stained cytologic smears permit to estimate the topographic localization of methylated regions in the nucleus. Co-localization analysis has shown that the deeply Giemsa-stained compacted heterochromatin domains have the same geographic distribution as the methyl-rich regions within each nucleus [73]. Therefore, aggressive myelomas should have a more complex chromatin structure with an increased number of darker and lighter areas, leading to a higher fractal dimension of the nuclear chromatin, as found in our study.

Indeed, the FD of MGG-stained nuclear chromatin showed to be an independent adverse prognostic factor for the overall survival of our patients. In a similar way, previous studies have demonstrated an association between a higher FD value of the nuclear chromatin and a worse outcome of patients with other neoplasias, such as malignant melanomas, squamous cell carcinomas of the oral cavity and larynx [14], [28]-[31].

This implies that the complexity of chromatin distribution contains important prognostic information which is independent of clinical variables, ISS stage, or relevant cytogenetic aberrations. In the present study, the frequency of cytogenetic abnormalities was low when compared to other reports [2], [3]. Technical problems, however, could have precluded the finding of some abnormalities.

The goodness-of-fit of the fractal dimension was also of independent prognostic relevance, but as a favorable factor. Thus a chromatin architecture closer to the "ideal fractal" was associated with a prolonged survival of the patient, as it has been shown previously for blasts of B precursor acute lymphatic leukemia [10].

Explanations for this finding are speculative at the moment. But it might be possible that the large number of genetic and epigenetic modifications in aggressive tumors could disturb the process of auto-organization of the nucleus to such an extent that the scale-free auto-similarity of chromatin structures is not as perfect as in less aggressive cases.

Our study revealed that both the fractal dimension and its goodness-of-fit permit to quantify DNA remodeling and methylation status in MGG-stained bone marrow smears of myeloma patients and therefore may be new and biologically relevant prognostic factors for this disease. A more detailed scientific validation of the texture analyses is necessary, of course. Data from genome-wide methylation or chromatin analyses should be compared with fractal data derived from digitalized images of routinely stained tumor smears or sections, in order to define better the equivalence between changes of the image texture and genome-wide biochemical chromatin changes.

Since there is a vast heterogeneity of molecular profiles among myeloma patients, detailed individual genomic evaluations for targeted therapies seem not to be helpful at the moment, as has been emphasized recently [74].

In this situation, a global evaluation of the nucleus, as presented in this investigation, could be interesting. This technique is simple, reproducible and unexpensive and may be applied to routine slides from the files, thus permitting retrospective studies without any additional costs. Therefore, we think it could be useful in daily routine practice in future. But since our study was based on a relatively small number of patients, it should, of course, be followed by confirmatory investigations based on more and new patients in different centers [75].

## References

[1] Leleu X, Genevieve F, Guieze R, Duhamel A, Andrieux J (2005). Irregular nuclear shape of bone marrow plasma cells defines a multiple myeloma subgroup related to hypodiploidy and to short survival.. Leukemia.

[2] Greipp PR, San Miguel J, Durie BG, Crowley JJ, Barlogie B (2005). International staging system for multiple myeloma.. J Clin Oncol.

[3] Tinguely M, Jenni B, Reineke T, Korol D, Kofler A (2007). Chromosomal translocations t(4;14), t(11;14) and proliferation rate stratify patients with mature plasma cell myelomas into groups with different survival probabilities - A molecular epidemiologic study on tissue microarrays.. Am J Surg Pathol.

[4] Ortega MM, Cunha AF, Albuquerque DM, Costa GL, De Souza CA (2008). Identification of new overexpressed genes related to cell proliferation, stimulation and apoptosis inhibition of plasma cells of multiple myeloma by Sage method.. Ann Oncol.

[5] Rajkumar SV, Buadi F (2007). Multiple myeloma: new staging systems for diagnosis, prognosis and response evaluation.. Best Pract Res Clin Haematol;.

[6] Goasguen JE, Zandecki M, Mathiot C, Scheiff JM, Bizet M (1999). Mature plasma cells as indicator of better prognosis in multiple myeloma. New methodology for the assessment of plasma cell morphology.. Leukemia Res.

[7] Genty V, El-Khoury V, Liautaud-Roger F, Dine G, Dufer J (2005). Nuclear chromatin patterns in 3 glucocorticoid-resistant RPMI 8226 human myeloma cell sub-lines: correlations with cell growth and immunological phenotype.. Cancer Biol Ther.

[8] Metze K, Adam RL, Kayser G, Kayser K (2010). Pathophysiology of cancer and the entropy concept, Model-Based Reasoning in Science and Technology.. Studies in Computational Intelligence 314,.

[9] Metze K, Oliveira GB, Pereira FG, Adam RL, Lorand-Metze I (2005). Spontaneous apoptosis in chronic lymphocytic leukemia is not an independent prognostic factor for stability of disease when compared with combined AgNOR and TTM scores.. Cell Oncology.

[10] Adam RL, Silva RC, Pereira FG, Leite NJ, Lorand-Metze I (2006). The fractal dimension of nuclear chromatin as a prognostic factor in acute precursor B lymphoblastic leukemia.. Cell Oncol.

[11] Montironi R, Scarpelli M, Lopez-Beltran A, Mazzucchelli R, Alberts D (2007). Chromatin phenotype karyometry can predict recurrence in papillary urothelial neoplasms of low malignant potential.. Cell Oncol.

[12] Metze K, Bedin V, Adam RL, Cintra ML, de Souza EM (2005). Parameters derived from the fast Fourier transform are predicitive for the recurrence of basal cell carcinoma. Cell.. Oncol.

[13] Nielsen B, Albregtsen F, Kildal W, Danielsen HE (2001). Prognostic classification of early ovarian cancer based on very low dimensionality adaptive texture feature vectors from cell nuclei from monolayers and histological sections.. Anal Cell Pathol.

[14] Bedin V, Adam RL, Sá BCS, Landman G, Metze K (2010). Fractal dimension is an independent prognostic factor for survival in melanoma.. BMC Cancer.

[15] Lorand-Metze I, Pereira FG, Costa FP, Metze K (2004). Proliferation in non-Hodgkin's lymphomas and its prognostic value related to staging parameters.. Cell Oncology.

[16] Losa GA (2009). The fractal geometry of life.. Riv Biol.

[17] Einstein AJ, Wu HS, Sanchez M, Gil J (1998). Fractal characterization of chromatin appearance for diagnosis in breast cytology.. J Pathol.

[18] Lopes R, Betrouni N (2009). Fractal and multifractal analysis: a review.. Med Image Anal.

[19] Rocha LB, Adam RL, Leite NJ, Metze K, Rossi MA (2008). Shannon's entropy and fractal dimension provide an objective account of bone tissue organization during calvarial bone regeneration.. Microsc Res Tech.

[20] Herreros FO, Cintra ML, Adam RL, de Moraes AM, Metze K (2007). Remodeling of the human dermis after application of salicylate silanol.. Arch Dermatol Res.

[21] Lorthois S, Cassot F (2010). Fractal analysis of vascular networks: insights from morphogenesis.. J Theor Biol.

[22] Dey P, Banik T (2011). Fractal dimension of chromatin texture of squamous intraepithelial lesions of cervix.. Diag Cytopathol.

[23] Ferreira RC, de Matos PS, Adam RL, Leite NJ, Metze K (2006). Application of the Minkowski-Bouligand fractal dimension for the differential diagnosis of thyroid follicular neoplasias.. Cell Oncol.

[24] Metze K, Soares A, Adam R, Araujo V, Altemani A (2008). Vessel remodelling during tumour progression of carcinoma ex pleomorphic adenoma.. Cell Oncol.

[25] Tambasco M, Magliocco AM (2008). Relationship between tumor grade and computed architectural complexity in breast cancer specimens.. Hum Pathol.

[26] Lieberman-Aiden E, Van Berkum NL, Williams L, Imakaev M, Ragoczy T (2009). Comprehensive mapping of long-range interactions reveals folding principles of the human genome.. Science.

[27] Bancaud A, Huet S, Daigle N, Mozziconacci J, Beaudouin J (2009). Molecular crowding affects diffusion and binding of nuclear proteins in heterochromatin and reveals the fractal organization of chromatin.. EMBO J.

[28] Metze K (2010). Fractal dimension of chromatin and cancer prognosis.. Epigenomics.

[29] Goutzanis L, Papadogeorgakis N, Pavlopoulos PM, Katti K, Petsinis V (2008). Nuclear fractal dimension as a prognostic factor in oral squamous cell carcinoma.. Oral Oncol.

[30] Mashiah A, Wolach O, Sandbank Uziel O, Raanani P, Lahav M (2008). Lymphoma and leukemia cells possess fractal dimensions that correlate with their biological features.. Acta Haematol.

[31] Delides A, Panayiotides I, Alegakis A, Kyroudi A, Banis C (2005). Fractal dimension as a prognostic factor for laryngeal carcinoma.. Anticancer Res.

[32] Nielsen B, Albregtsen F, Danielsen HE, Losa GA, Merlini D, Nonnenmacher TF, Weibel ER (2005). Fractal Analysis of Monolayer Cell Nuclei from Two Different Prognostic Classes of Early Ovarian Cancer.. Fractals in Biol and Med.

[33] Irinopoulou T, Rigaut JP, Benson MC (1993). Toward objective prognostic grading of prostatic carcinoma using image analysis.. Anal Quant Cytol Histol.

[34] The International Myeloma Working Group (2003). Criteria for the classification of monoclonal gammopathies, multiple myeloma and related disorders: a report of the International Myeloma Working Group.. Br J Haematol.

[35] Brigaudeau C, Gachard N, Clay D, Fixe P, Rouzier E (1996). Miniaturized method for the karyotype analysis of bone marrow or blood samples in hematological malignances. Hematol.. Cell Ther.

[36] Maiolino A, Hungria VT, Oliveira-Duarte G, Oliveira LC, Mercante DR (2008). Thalidomide + Dexamethasone as Maintenance after Single Autologous Stem Cell Transplantation Improves Progression-Free Survival (PFS) in Advanced Multiple Myeloma. A Prospective Brazilian Randomized Trial.. Blood.

[37] Metze K (2009). Pitfalls in prognostic factor studies.. J Cutan Pathol.

[38] Metze K (2008). Dichotomization of continuous data-a pitfall in prognostic factor studies.. Pathol Res Pract.

[39] Dubuc B, Quiniou JF, Roques-Carmes C, Tricot C, Zucker SW (1989). Evaluating the fractal dimension of profiles.. Physical Reviews A.

[40] Albregtsen F (2009). How to calculate the goodness-of-fit of a fractal dimension.. Cell Oncol.

[41] Metze K, Lorand-Metze I, Leite NJ, Adam RL (2009). Goodness-of-fit of the fractal dimension as a prognostic factor.. Cell Oncol.

[42] Metze K, Lobo AM, Lorand-Metze I (2000). Nucleus organizer regions (AgNORs) and total tumor mass are independent prognostic parameters for treatment-free period in chronic lymphocytic leukemia.. Inter J Cancer.

[43] Rybka MO, Cintra ML, de Souza EM, Metze K (2008). Density of dendritic cells around basal cell carcinomas is related to tumor size, anatomical site and stromal characteristics, and might be responsible for the response to topical therapy.. Int J Dermatol.

[44] Renshaw C, Ketley N, Møller H, Davies EA (2010). Trends in the incidence and survival of multiple myeloma in South East England 1985-2004.. BMC Cancer.

[45] Hungria VT, Maiolino A, Martinez G, Colleoni GW, Coelho EO (2008). Confirmation of the utility of the International Staging System and identification of a unique pattern of disease in Brazilian patients with multiple myeloma.. Haematologica.

[46] Rego MFN, Pinheiro GS, Metze K, Lorand-Metze I (2003). Acute leukemias in Piauí: comparison with features observed in other regions of Brazil.. Braz J Med Biol Res.

[47] Pagnano KBB, Silveira RA, Nardinelli, Mello M, De Souza CA (2008). Outcome of patients with chronic myeloid leukemia with T315l BCR-ABL mutation.. Haematologica.

[48] Lorand-Metze I, Pinheiro MP, Ribeiro E, de Paula EV, Metze K (2004). Factors influencing survival in myelodysplastic sybdromes in a Brazilian population: Comparison of FAB and WHO classifications.. Leuk Res.

[49] Pereira FG, Metze K, Costa FPS, Lima CSP, Lorand-Metze I (2006). Phenotypic quantitative features of patients with acute myeloid leukemia.. Neoplasma.

[50] Lopes LF, Lorand-Metze I, Niero-Melo L, Tone LG, Velloso E (2002). The Brazilian pediatric myelodysplastic cooperative group strategies: are they relevant to improve educational approach and correct diagnosis?. Leuk Res.

[51] Anagnostopoulos A, Gika D, Symeonidis A, Zervas K, Pouli A (2005). Multiple myeloma in elderly patients: prognostic factors and outcome.. Eur J Haematol.

[52] Jin Lee W, Hoppin JA, Blair A, Luvin H, Dosemeci M (2004). Cancer Incidence among Pesticide Applicators Exposed to Alachlor in the Agricultural Health Study.. Am J Epidemiol.

[53] Faria NMX, Fassa AG, Facchini LA (2007). Pesticides poisoning in Brazil: the official notification system and challenges to conducting epidemiological studies. Ciênc.. saúde coletiva.

[54] Gebara AB, Ciscato CH, Monteiro SH, Souza GS (2011). Pesticide Residues in some Commodities: Dietary Risk for Children.. Bull Environ Contam Toxicol.Publish on line April.

[55] Kayser K, Kayser G, Metze K (2007). The concept of structural entropy in tissue-based diagnosis.. Anal Quant Cytol Histol.

[56] Jondet M, Agoli-Agbo R, Dehennin L (2010). Automatic measurement of epithelium differentiation and classification of cervical intraneoplasia by computerized image analysis.. Diagn Pathol.

[57] Kayser K, Hoshang SA, Metze K, Goldmann T, Vollmer E (2008). Texture- and object-related automated information analysis in histological still images of various organs.. Anal Quant Cytol Histol.

[58] Losa GA, Graber R, Baumann G, Nonnenmacher TF (1998). Steroid Hormones Modify Nuclear Heterochromatin Structure and Plasma Membrane Enzyme of MCF-7 Cells. A Combined Fractal, Electron Microscopic and Enzymatic Analysis.. Eur J Histochem.

[59] Losa GA, Castelli C (2005). Nuclear patterns of human breast cancer cells during apoptosis: characterization by fractal dimension and co-occurrence matrix Statistics.. Cell Tissue Res.

[60] Nielsen B, Albregtsen F, Danielsen HE, Losa GA, Merlini D, Nonnenmacher TF,  Weibel ER (2005). Using Fractal Signature Vectors and Lacunarity Class Distance Matrices to Extract New Adaptive Feature from Cell Nuclei.. Fractals in Biol and Med.

[61] Metze K, Adam RL, Vido JR, Lorand-Metze I (2009). The influence of staining characteristics on nuclear texture features in cytology.. Anal Quant Cytol Histol.

[62] Metze K, Adam RL (2009). Intrinsic problems of the nuclear shape factor analysis.. Dis Colon Rectum.

[63] Metze K, Adam RL, Ferreira RC (2010). Robust variables in texture analysis. Pathology.. 2010;.

[64] Mandelbrot BB (1975). Stochastic models for the Earth's relief, the shape and the fractal dimension of the coastlines, and the number-area rule for islands.. Proc Natl Acad Sci U S A.

[65] Cattani C, Gaetano P (2011). Complexity on acute myeloid leukemia mRNA transcript variant.. Mathematical Problems in Engineering.

[66] Aon MA, Roussel MR, Cortassa S, O'Rourke B, Murray DB (2008). The Scale-Free Dynamics of Eukaryotic Cells Plos ONE;.

[67] Thamrin C, Stern G, Frey U (2010). Fractals for physicians.. Paediatr Respir Rev.

[68] McNally JG, Mazza D (2010). Fractal geometry in the nucleus.. EMBO J;.

[69] Wolfram S (2002). A new kind of science.. Ed Wolfram Media Inc.

[70] Raab MS, Podar K, Breitkreutz I, Richardson PG, Anderson KC (2009). Multiple myeloma.. Lancet.

[71] De Bruyne E, Bos TJ, Asosingh K, Vande Broek I, Menu E (2008). Epigenetic Silencing of theTetraspanin CD9 during Disease Progression in Multiple Myeloma Cells and Correlation with Survival.. Clin Cancer Res.

[72] Bollati V, Fabris S, Pegoraro V, Ronchetti D, Mosca L (2009). Differential repetitive DNA methylation in multiple myeloma molecular subgroups.. Carcinogenesis.

[73] de Capoa A, Febbo FR, Giovannelli F, Niveleau A, Zardo G (1999). Reduced levels of poly(ADP-ribosyl)ation result in chromatin compaction and hypermethylation as shown by cell-by-cell computer-assisted quantitative analysis.. FASEB J.

[74] Avet-Loiseau H, Magrangeas F, Moreau P, Attal M, Facon T (2011). Molecular Heterogeneity of Multiple Myeloma: Pathogenesis, Prognosis, and Therapeutic Implications.. J Clin Oncol.

[75] Elston LB, Sueiro FA, Cavalcanti JN, Metze K (2009). The importance of the mitotic index as a prognostic factor for survival of canine cutaneous mast cell tumors: a validation study.. Vet Pathol.

